# Melatonin Ameliorates the Progression of Alzheimer's Disease by Inducing TFEB Nuclear Translocation, Promoting Mitophagy, and Regulating NLRP3 Inflammasome Activity

**DOI:** 10.1155/2022/8099459

**Published:** 2022-08-09

**Authors:** Li Fan, Xie Zhaohong, Wang Xiangxue, Xu Yingying, Zhang Xiao, Zhou Xiaoyan, Yan Jieke, Lai Chao

**Affiliations:** Department of Neurology, The Second Hospital of Shandong University, Shandong University, Jinan 250033, China

## Abstract

**Background:**

The NLRP3 inflammasome is overactivated in the brains of APP/PS1 transgenic mice and AD patients, and mitophagy has an obvious negative regulatory role on NLRP3 inflammasome activation. The protective effect of melatonin in AD may be related to the regulation of mitophagy and NLRP3 inflammasome activity. TFEB plays a critical role in maintaining autophagy/mitophagy. Studies have found that TFEB plays a protective role in AD.

**Methods:**

APP/PS1 transgenic mice were given melatonin in their drinking water for 3 months. Compared with mice without melatonin treatment, the mice given melatonin showed changes in the following features: (1) cognitive function, (2) mitophagy-related proteins in the brain, (3) ROS, (4) NLRP3 inflammasome and related proteins and the concentrations of inflammatory cytokines, and (5) A*β* deposition. In *in vitro* experiments, effects of melatonin on mitophagy, NLRP3 inflammasome activity, and TFEB in SH-SY5Y cells with A*β*_25-35_ were observed. TFEB knockdown was implemented in combination with A*β*_25-35_ and melatonin treatment, and the expressions of TFEB, Parkin, p62, IL-1*β*, caspase-1, ROS, and IL-18 were explored.

**Results:**

Melatonin improved cognitive function in APP/PS1 transgenic mice and decreased ROS and senile plaques. Melatonin promoted mitophagy in SH-SY5Y cells with A*β*_25-35_ and APP/PS1 transgenic mice. NLRP3 inflammasome activity was inhibited, and the concentrations of IL-18 and IL-1*β*were clearly reduced. Compared with C57/BL6J mice, the amount of TFEB in the brain nucleus of APP/PS1 transgenic mice was decreased. Melatonin treatment increased the nuclear translocation of TFEB in SH-SY5Y cells. TFEB knockout was implemented in combination with A*β*_25-35_ and MT treatment; the expressions of Parkin, p62, caspase-1, IL-1*β*, IL-18, and ROS were accelerated.

**Conclusions:**

Melatonin promotes mitophagy by inducing TFEB nuclear translocation, downregulates NLRP3 inflammasome activation, and exerts protective effects in SH-SY5Y cells and APP/PS1 transgenic mice.

## 1. Background

Alzheimer's disease (AD) is one of the most common diseases closely related to age, is also known as senile dementia, occurs in the elderly and presenile patients, and is characterized by behavioural disorder and progressive cognitive impairment. To date, the pathogenesis and aetiology of AD remain unknown, and there is no effective treatment for AD. Hence, further research on the pathogenesis and aetiology of AD is urgently needed to aid the identification of treatment methods for AD treatment.

A persistent excessive inflammatory response plays a key role in the pathophysiological mechanisms of AD [1]. The microglial-mediated inflammatory response is a focus of AD research. Microglia play a vital role in A*β* clearance.

Pattern-recognition receptors (PRRs) have the capacity to recognize foreign stimuli and sense damage-specific proteins in the body. NLRs (NOD-like receptors) are PRRs that are localized in the cell and can recruit precursors of procaspase-1 directly or through apoptosis-associated speck-like protein containing a CARD (ASC) to form a protein complex of inflammasomes. The assembly of the inflammasome can convert procaspase-1 into caspase-1, which converts pro-IL-18 and IL-1*β* into mature IL-18 and IL-1*β* in turn [2]. The best characterized inflammasome is the NLRP3 inflammasome. Mitochondria are essential for NLRP3 inflammasome activation, and signals from abnormal mitochondrial function, such as phospholipid externalization, oxidized mtDNA, and ROS, can intervene in the activation of NLRP3 [3]. Kirchmeyer et al. [4] found that caspase-1, ASC, and NLRP3 were in brain microglia, indicating that the activation of the NLRP3 inflammasome in the brain is mainly in microglia. A*β* can stimulate IL-1*β* production in microglia [5]. IL-1*β* in AD patients' cerebrospinal fluid, brain tissue, and peripheral blood is sharply accelerated [6]. Caspase-1 and IL-1*β* are highly expressed in brain tissues or neurons of AD transgenic mice treated with A*β* [7], especially around A*β* plaques [8]. IL-1*β* plays a key role in the pathophysiology of AD, and is a main effector of the activation in the NLRP3 inflammasome. Halle et al. [9] found that A*β* promotes microglial lysosome destruction and cathepsin B release, which activates the NLRP3 inflammasome and further leads to microglial secretion of IL-1*β*, inducing an inflammatory response and continuous overactivation of microglia via downstream signal transduction pathways. These studies suggest that the NLRP3 inflammasome is overactivated and is the core mechanism of inflammation in AD.

Overactivation of the NLRP3 inflammasome is related to the mitochondrial damage and abnormal mitophagy. Mitochondria play an important role in eukaryotic cells by participating in biological oxidation and energy conversion and participate in multiple biological processes, such as intracellular homeostasis, proliferation, ageing, and cell death. Asymmetric division of mitochondria can lead to weakening or disappearance of mitochondrial membrane potential or depolarization of mitochondria; various stimuli both *in vitro* and *in vivo*, such as A*β* oligomers, can also cause pathological depolarization of mitochondria. These depolarized mitochondria can be recycled through mitochondrial fusion or through selective autophagy, which is called mitophagy. When the mitochondrial membrane is damaged, PINK1 recruits Parkin into mitochondria to facilitate mitophagy. This decrease in mitochondrial clearance can lead to the accumulation of damaged mitochondria, causing mitochondrial dysfunction, and eventually leading to neurodegenerative diseases. Mitophagy plays a vital role in the pathogenesis of AD, and the number of normal mitochondria in the hippocampal neurons of AD patients is significantly reduced.

Mitochondrial injury plays a key role in NLRP3 inflammasome activation, and as an important mechanism of clearing damaged mitochondria, mitophagy plays a key regulatory role in NLRP3 inflammasome activation. Zhong et al. discovered that when cells undergo inflammatory damage, the increased P62 content is transferred to damaged mitochondria, where Parkin ubiquitination induces mitochondrial autophagy [10]. Consistent with this finding, Kim et al. also observed an increase in P62 in NLRP3 inflammasome-activated cells and transfer of P62 to impaired mitochondria to induce mitochondrial autophagy [11].

Melatonin (N-acetyl-5-methoxy-tryptamine), a neurohormone from the pineal gland, participates in the regulation of various physiological functions. In disease and ageing, decreased melatonin levels lead to abnormal physiological functions. Melatonin reduction in elderly individuals may itself be an important factor leading to neurodegenerative disease in the elderly and is considered to be one of the main causes of AD [12]. Melatonin can prevent the increase of lipid peroxidation, free radical production, oxidative protein damage, and oxidative DNA damage in AD and decrease ATP production. Melatonin plays a protective role by improving mitophagy, which has been demonstrated in models of many diseases other than AD. Ma et al. [13] found in animal models of atherosclerosis that melatonin prevents atherosclerosis progression by inducing Parkin signalling pathway-mediated mitophagy and attenuating NLRP3 inflammasome activation. Cao et al. [14] found that mitophagy mediated by melatonin protected the early brain injury after subarachnoid haemorrhage by inhibiting NLRP3 inflammasome activation. However, the effect of melatonin on mitophagy in AD has not been reported.

Autophagy/mitophagy is regulated by a series of complex signalling molecules, among which transcription factor EB (TFEB) is the main regulator. TFEB is a member of the MiT transcription factor family that promotes mitophagy via the regulation of autophagosome-lysosomal fusion and autophagosome formation [15]. TFEB, a transcription factor with a BHLH-ZIP structure [16], binds to promoter motifs or CLEAR elements to regulate lysosomal gene expression [17]. Normally, TFEB is located in the cytoplasm. Under stress conditions, such as starvation and lysosomal dysfunction, TFEB can be translocatesd to the nucleus to facilitate the transcription of target genes. TFEB-mediated mitophagy has been found to improve the pathological changes and cognitive function of AD [18].

In this article, we observed the effects of melatonin on the cognitive function of APP/PS1 transgenic mouse models, mitophagy, the NLRP3 inflammasome and related regulatory proteins, and TFEB.

## 2. Methods

### 2.1. Animals and Drug Treatment

The experimental animals were C57/BL6J mice and APP/PS1 transgenic mice with C57/BL6J as the genetic background. All 30 mice were male to eliminate possible gender influence. The experimental animals were obtained from Beijing HFK Bio-Technology Co., Ltd.

The experimental animals were distributed into 3 groups with 10 mice in each group. The mice in each group were fed from 6 months to 9 months of age. C57/BL6J mice were fed double steamed water; APP/PS1 transgenic mice in the placebo group were fed double steamed water. APP/PS1 transgenic mice in the melatonin intervention group were fed double steamed water plus melatonin. The mice drank 5 mL water on average every day, and the estimated daily intake of melatonin was approximately 0.5 mg. All mice were subjected to a water maze test. The mice in each group were randomly distributed into two groups with 5 mice in each group. One group was used for brain harvesting by cardiac perfusion, and the other group was used for fresh brain tissue harvesting.

### 2.2. Morris Water Maze

The Morris water maze test was carried out to evaluate the spatial memory and learning of mice. The same conditions were used around the water maze to prevent the influence of environmental changes on the memory reference of the mice and to prevent interference from other objects and the video tracking system of the experimenters. Lamps were placed around the water maze to provide light, and the water temperature was controlled at 22 ± 1°C. The first day was the adaptation period for the mice. The mice to be tested were successively put into the water maze without a platform for approximately 1 minute of swimming practice. Days 2-6 of the water maze were the learning period, which was mainly used to evaluate the learning ability of the mice. At this stage, the platform was put into the water maze in the SW (southwest) direction. The camera was set 2 m above the pool, and software was used to record the mouse position, swimming path, and time required to reach the platform position (escape latency). The seventh day was the exploratory period. In the exploration experiment, the platform was moved away, and the mice were introduced into the water in a new direction, NE (northeast). The mice needed to find the original platform location by memory. The recording time was 60 s, and the time spent in the target quadrant and the number of platform location crosses were recorded.

### 2.3. Cell Culture and Reagents

The human neuroblastoma cell line SH-SY5Y was from the Cell Bank of the Chinese Academy of Sciences and was cultivated in DMEM with 15% FBS (Gibco, Rockville, USA), 100 U/mL penicillin, and100 g/mL streptomycin. Cells were cultured under the conditions of 5% CO_2_, 37°C, and high humidity.

### 2.4. Extraction of Total Proteins and Cells from Brain Tissues

Brain tissue were quickly frozen and stored at −80°C. Ice-cold RIPA lysis buffer (Beyotime, Shanghai, China) was used for homogenizing brain samples. After centrifugation at 12,000 × g at 4°C for 20 minutes, western blotting was performed on the supernatant.

After digestion and centrifugation, the cultured cells were cultured in 6 mm petri dishes. The cells was prepared into a single cell suspension with 1x PBS (1 mL) and placed on ice. Then, an appropriate amount of protein lysate was added. After trituration and denaturation at 100°C for 5 h, the cells were lysed completely. The protein concentration was quantified by 5 *μ*L aliquot, and the remaining protein was stored at -20°C.

### 2.5. Western Immunoblotting Analyses

Proteins were obtained by RIPA lysis buffer containing fresh protease and phosphate inhibitor mixture and boiled for denaturation. Protein concentration was determined by BCA protein assay. Cell lysate was then prepared for western blotting using a 10% polyacrylamide gel and 30 *μ*g of protein. After electrical transfer and blocking with 5% BSA, the membrane was incubated with primary antibodies at 4°C overnight. Antibodies against *β*-actin (A5441) were obtained from Sigma–Aldrich; antibodies against TFEB (ab270604), NLRP3 (ab263899), PINK1 (ab23707), and Parkin (ab77924) were purchased from Abcam; and antibodies against GAPDH (SC-365062), caspase-1 (SC-56036), and P62 (SC-48402) were obtained from Santa Cruz Biotechnology.

### 2.6. Real-Time Quantitative PCR

Total RNA was obtained via a TRIzol Kit. PrimeScript RT Kit (Takara, Japan) was used for preparing the cDNA. SYBR Green was used for qRT-PCR, and the primers are listed in Table 1.

### 2.7. Transfection

The pcDNA3.1-TFEB plasmid and pcDNA3.1 (negative control) were transfected into cells by Lipofectamine 3000 (Invitrogen, Carlsbad, USA). Lentiviral shRNA interference vectors targeting TFEB (shTFEB) and negative control vector (short hairpin RNA [shRNA]) were obtained from Hanbio Biotechnology (Shanghai, China). The TFEB shRNAs were as follows: shTFEB (forward), 5′-CCGGCCCACTTTGGTGCTAATAGCTCTCGAGAGCTATTAGCACCAAAGTGGGTTTTTG-3′; shTFEB (reverse), 5′-AATTCAAAAACCCACTTTGGTGCTAATAGCTCTCGAGAGCTATTAGCACCAAAGTGGG-3′.

### 2.8. Immunofluorescence

Cells were transfected with the pcDNA3.1-TFEB plasmid or treated with MT and then inoculated on glass slides overnight. The cells were fixed with 4% paraformaldehyde for 5 min and incubated with the primary antibody overnight at 4°C. The next day, the cells were incubated with the secondary antibody for 2 h. After 10 min of DAPI staining, the samples were then imaged by a microscope (LSM800, Carl Zeiss).

### 2.9. Reactive Oxygen Species Assay

The level of ROS in SH-SY5Y cells were examined by a 2′7′-dichlorofluorescin diacetate (DCFH-DA) assay kit. 1 × 10^6^ cells/well were inoculated in a 6-well plate. The cells were suspended in DCFH-DA (200 *μ*L) at 37°C in the dark for 20 minutes. After washing with PBS twice, the fluorescence intensity of cells was measured by a microplate reader (Cytation 5, America).

### 2.10. Subcellular Fractionation

Subcellular fractions (cytosolic and nuclear) were isolated from cells as described with modifications [19]. Briefly, cells were lysed in a NP-40 lysis buffer with EDTA (0.5 mM), NaCl (150 mM), Tris-HCl (20 mM, pH 7.9), and NP-40 (0.5%) with phosphatase and protease inhibitors. The lysed cells were placed on ice for 15 min and then centrifuged at 2,000 × g for 5 min. The corresponding pellets representing the nuclear fractions were washed once in an NP-40-containing lysis buffer and sonicated in a nuclear lysis buffer (450 mM NaCl, 20 mM Tris-HCl (pH 7.4), 0.5% Triton X-100, 0.1% SDS, and 0.5 mM EDTA). The lysates were centrifuged at 12,000 × g for 15 min to acquire the nuclear and cytosolic fractions.

### 2.11. Statistical Analysis

The data were analysed by GraphPad Prism software and presented as the mean ± SD. One-way ANOVA was used for comparisons among different groups. Student's *t* test was used for comparisons between two groups. All experiments were repeated at least three times. *P* < 0.05 was defined as a statistical significance.

## 3. Results

### 3.1. Melatonin Can Improve Cognitive Function and Decline A*β* Deposition in APP/PS1 Transgenic Mice

APP/PS1 transgenic mice were given melatonin through drinking water for 3 months (from 9 to 12 months, 0.5 mg melatonin daily). Compared with the placebo control APP/PS1 transgenic mice, the escape latency of the melatonin intervention group was shortened (Figure 1(a)) and significantly different on Day 5 (Figure 1(b)), with an increased number of platform crossings (Figure 1(c)) and a longer time in the target quadrant (Figure 1(d)). There was no obvious difference in swimming speed (Figure 1(e)). Thioflavin staining was used to detect senile plaques. The results showed that the number of senile plaques in the cerebral cortex and hippocampus of APP/PS1 transgenic mice in the melatonin intervention group was significantly reduced compared with that of APP/PS1 transgenic mice in the placebo control group (Figures 1(f) and 1(g)).

### 3.2. Melatonin Promoted Mitophagy and Inhibited NLRP3 Inflammasome Activity in APP/PS1 Transgenic Mice

After 3 months of melatonin intervention, western blot analysis showed that compared with the placebo control group APP/PS1 transgenic mice, the levels of the mitophagy-related protein PINK1 were increased in the brains of APP/PS1 transgenic mice in the melatonin intervention group, while the levels of Parkin and P62 were decreased. The levels of caspase-1 and NLRP3 inflammasome components were significantly decreased (Figure 2(a)). The expression of PINK1 and LC3 in frozen brain tissue sections was observed by immunofluorescence. The levels of PINK1 and LC3 were increased in the melatonin intervention group (Figure 2(b)). ROS levels in the APP/PS1 transgenic mice were dramatically reduced in the melatonin intervention group (Figure 2(c)). The levels of IL-18, IL-6, and IL-1*β* were notably decreased according to real-time quantitative PCR (Figure 2(d)). These results suggest that melatonin can promote mitophagy and inhibit NLRP3 inflammasome activity.

### 3.3. Melatonin Improved Mitophagy and Inhibited the NLRP3 Inflammasome In Vitro

After pretreatment with melatonin (10 *μ*M), the levels of the mitophagy-related proteins caspase-1, P62, and Parkin were decreased in SH-SY5Y cells treated with A*β*_25-35_ (Figure 3(a)). Colocalization of PINK1 and LC3 was detected by immunofluorescence. The colocalization of PINK1 and LC3 was increased in the melatonin-pretreated group (Figure 3(b)). ROS levels were clearly reduced in the melatonin intervention group (Figure 3(c)). The levels of IL-1*β* and IL-18 were significantly decreased, as shown by real-time quantitative PCR (Figure 3(d)). With the addition of the autophagy inhibitor hydroxychloroquine (HCQ-10 *μ*M), ROS levels significantly increased (Figure 3(e)). The levels of IL-18 and IL-1 were notably increased (Figure 3(f)).

### 3.4. Melatonin Increased the Amount of TFEB in the Brain Nucleus of APP/PS1 Transgenic Mice, and TFEB Promoted Mitophagy and Alleviated the A*β*-Induced Inflammatory Response In Vitro

TFEB levels in the brain nucleus of APP/PS1 transgenic mice were significantly reduced in APP/PS1 transgenic mice (Figure 4(a)). With the addition of TFEB, the levels of the mitophagy-related proteins caspase-1, P62, and Parkin were decreased in SH-SY5Y cells with A*β*_25-35_ (Figure 4(b)). After overexpressing TFEB in SH-SY5Y cells and treating them with A*β*_25-35_, the colocalization of LC3 and PINK1 increased, as detected by immunofluorescence, suggesting enhanced mitophagy (Figure 4(c)). With the addition of TFEB, ROS levels significantly decreased (Figure 4(d)). The levels of IL-18 and IL-1 were significantly decreased (Figure 4(e)).

### 3.5. Melatonin Alleviated the Toxic Effects of A*β* by Promoting TFEB Nuclear Translocation

After melatonin treatment, an increase in the nuclear translocation of TFEB was detected by immunofluorescence in SH-SY5Y cells (Figure 5(a)). The level of TFEB in the nucleus was significantly increased after treatment with melatonin, as detected by western blotting (Figure 5(b)). shRNA knockdown of TFEB was implemented in combination with A*β*_25-35_ and MT treatment, and the expression of Parkin, p62, and caspase-1 increased (Figure 5(c)). The level of ROS increased (Figure 5(d)). The expression of IL-18 and IL-1*β* also increased (Figure 5(e)).

## 4. Discussion

Mitochondrial damage is an early feature of AD and causes pathological changes in A*β* and Tau [20]. Mitophagy is a normal process in which cells detect and remove damaged mitochondria, and it is very important for maintaining a healthy mitochondrial pool and the healthy survival of neurons. Mitophagy disorders lead to the accumulation of dysfunctional mitochondria in neurons, causing inflammation and promoting the progression of AD. The NLRP3 inflammasome is the core factor underlying AD inflammation, and excessive activation of the NLRP3 inflammasome is related to the mitochondrial damage and abnormal mitochondrial autophagy function. After mitochondrial injury, increased ROS production, mitochondrial DNA release, NLRP3 translocation to mitochondria, increased cardiolipin in the mitochondrial intima, etc., can induce the NLRP3 inflammasome and promote the activation and maturation of the interleukins IL-18 and IL-1*β*, leading to downstream inflammatory reactions and cell damage. Mitophagy can restrain the activation of the NLRP3 inflammasome. Mitophagy can inhibit NLRP3 inflammasome activation by scavenging ROS [21].

Melatonin is widely distributed in organisms and has antioxidative, antiageing, antiapoptotic, and other effects. Many basic and clinical studies have confirmed the protective effect of melatonin on AD. Previous studies have found that melatonin protects against AD by reducing A*β* production, alleviating A*β* toxicity, and regulating the expression of senescence-related genes. Intracellular oxidative damage is mainly caused by reactive oxygen species (ROS) produced in mitochondria [22]. The melatonin concentration in mitochondria is significantly higher than that in other organelles or cells [23]. Mitochondrial membranes contain transporters that help mitochondria rapidly absorb melatonin against a concentration gradient [24]. Mitochondria originate from bacteria that produce melatonin. Mitochondria are thought to produce melatonin [25]. Studies have shown that melatonin can improve mitophagy and inhibit NLRP3 inflammasome activation in animal models of subarachnoid haemorrhage and atherosclerosis. In macrophages cultured in vitro, oxidation-modified LDL stimulation can increase ROS production and lead to NLRP3 inflammasome activation, while melatonin treatment can reduce ROS production and inhibit NLRP3 inflammasome activation. However, there are few studies on the effect of melatonin on mitophagy in AD. In this study, we used oral melatonin to treat APP/PS1 transgenic mice and confirmed the protective role of melatonin in AD by water maze tests and assessment of A*β* deposition and soluble A*β*40 and A*β*42 concentrations. By detecting the levels of mitophagy and NLRP3 inflammasome-related proteins and inflammatory factors, we observed mitophagy disorder and excessive activation of the NLRP3 inflammasome in APP/PS1 transgenic mice, confirming that melatonin can improve mitophagy and inhibit NLRP3 inflammasome activity in AD animal models.

In this study, the specific mechanism by which melatonin promotes mitophagy in AD was further explored. Lysosomes are key in maintaining normal autophagy [26]. The autophagy–lysosome pathway is involved in regulating A*β* metabolism and Tau protein degradation, and there is obvious autophagy–lysosome pathway dysfunction in AD [27]. TFEB, a major regulator discovered in recent years, plays a key role in autophagy/mitophagy [28]. miR-128, an upregulated microRNA, is present in the hippocampus and monocytes of AD patients. miR-128 can downregulate TFEB, suggesting the presence of endogenous TFEB abnormalities in AD [29]. In multiple AD mouse models with A*β* and Tau pathology, the enhancement of the ALP expression by exogenous TFEB has been demonstrated to significantly reduce A*β* and Tau pathological changes, improve cognitive impairment, upregulate PINK1, and enhance autophagy/mitophagy [30]. Based on the above findings, we hypothesized that the mechanism by which melatonin promotes mitophagy in AD may be related to TFEB. In this study, we found that overexpression of TFEB improved mitochondrial autophagy, alleviated mitochondrial damage, and antagonized the cytotoxic effects of A*β* in AD cells, demonstrating that exogenously induced TFEB expression plays a protective role in AD. In animal models, TFEB was found to be reduced in neuron nuclei in AD mouse brain tissue, suggesting inadequate TFEB function and confirming the presence of endogenous TFEB abnormalities in AD. In vitro experiments showed that melatonin can promote TFEB entry into the nucleus and improve mitophagy in AD.

This study confirmed the protective effect of melatonin in AD and found that the protective mechanism was related to the regulation of TFEB and the promotion of mitophagy, providing more evidence for the application of melatonin in the treatment of AD. TFEB intervention may become another potentially promising target for the treatment of AD.

## 5. Conclusions

Mitophagy disorder, overactivity of the NLRP3 inflammasome, and reduced TFEB content in the nucleus were found in APP/PS1 mouse brain tissue. Melatonin promotes mitophagy by inducing TFEB nuclear translocation, inhibits NLRP3 inflammasome activation, and exerts protective effects in AD.

## Figures and Tables

**Figure 1:** (a) Compared with placebo control APP/PS1 transgenic mice, the escape latency of the melatonin (MT) intervention group was shortened. (b) The escape latency was significantly different on day 5. (c) Compared with placebo control APP/PS1 transgenic mice, the number of platform crossings significantly increased in the MT intervention group. (d) The time in the target quadrant of the MT intervention group was significantly increased. (e) There was no significant statistical difference in swimming speed between the placebo control and MT intervention groups. (f) The number of senile plaques in the cerebral cortex was measured by thioflavin sulfur staining in APP/PS1 transgenic mice with TM treatment. The relative plaque burden ratio is shown on the left. (g) The number of senile plaques in the hippocampus was measured by thioflavin sulfur staining in APP/PS1 transgenic mice with TM treatment. The relative plaque burden ratio is shown on the left. *n* = 5 in each group. Data are presented as mean ± SEM. ^∗^*P* < 0.05; ^∗∗^*P* < 0.01; ^∗∗∗^*P* < 0.001.

**Figure 2:** (a) The levels of mitophagy-related proteins PINK1, Parkin, and p62 and the inflammasome-related protein caspase-1 and NLRP3 were detected by western blotting between placebo control and MT intervention groups. (b) Immunofluorescence method was used to detect the mitophagy-related proteins PINK1 and LC3. (c) The oxidative activated oxygen (ROS) of animal tissue was detected by luminol chemiluminescence kit between placebo control and MT intervention groups. (d) Expression of IL-1*β*, IL-6, and IL-18 mRNA was detected by qRT-PCR between placebo control and MT intervention groups. Data are presented as mean ± SEM. ^∗^*P* < 0.05; ^∗∗^*P* < 0.01; ^∗∗∗^*P* < 0.001.

**Figure 3:** The AD cell model was constructed in SH-SY5Y cells with A*β*_25-35_ treatment. (a) The levels of mitophagy-related proteins Parkin and p62 and the inflammasome-related protein caspase-1 were detected by western blotting with the MT treatment. (b) The colocalization between LC3 and PINK1 was detected by immunofluorescence with the MT treatment. (c) The lever of ROS was detected by luminol chemiluminescence kit with the MT treatment. (d) Expression of IL-1*β* and IL-18 mRNA was detected by qRT-PCR with the MT treatment. (e) Combined with MT and hydroxychloroquine (HCQ), the lever of ROS was detected by the luminol chemiluminescence kit. (f) Combined with MT and HCQ, the expression of IL-1*β* and IL-18 mRNA was detected by qRT-PCR. Data are presented as mean ± SEM. ^∗^*P* < 0.05; ^∗∗^*P* < 0.01; ^∗∗∗^*P* < 0.001.

**Figure 4:** (a) Western blotting analysis of the expression of TFEB in nucleus was performed in APP/PS1 transgenic mice. (b) SH-SY5Y cells overexpressing TFEB were treated with a combination of A*β*25-35, and the expressions of TFEB, Parkin, p62, and caspase-1 were detected by western blotting. (c) SH-SY5Y cells overexpressing TFEB were treated with a combination of A*β*25-35, and the colocalization between LC3 and PINK1 was detected by immunofluorescence. (d) SH-SY5Y cells overexpressing TFEB were treated with a combination of A*β*25-35, and the oxidative activated oxygen (ROS) was detected by luminol chemiluminescence kit. (e) SH-SY5Y cells overexpressing TFEB were treated with a combination of A*β*25-35, and the expression of IL-1*β* and IL-18 was analysed. Data are presented as mean ± SEM. ^∗^*P* < 0.05; ^∗∗^*P* < 0.01; ^∗∗∗^*P* < 0.001.

**Figure 5:** (a) Immunofluorescence analysis of the nuclear translocation of TFEB in SH-SY5Y cells incubated with MT. (b) Western blotting analysis of the nuclear translocation of TFEB in SH-SY5Y cells incubated with MT. (c) shRNA knockdown of TFEB was performed in combination with A*β*25-35 and MT treatment, and the expressions of TFEB, Parkin, p62, and caspase-1 were detected by western blotting. (d) shRNA knockdown of TFEB was performed in combination with A*β*25-35 and MT treatment, and the lever of ROS was detected by luminol chemiluminescence kit. (e) shRNA knockdown of TFEB was performed in combination with A*β*25-35 and MT treatment, and the expression of IL-1*β* and IL-18 was analysed. Data are presented as mean ± SEM. ^∗^*P* < 0.05; ^∗∗^*P* < 0.01; ^∗∗∗^*P* < 0.001.

**Table 1:** Primers for real-time quantitative PCR.

	Forward	Reverse
Mouse *β*-actin	GGCTGTATTCCCCTCCATCG	CCAGTTGGTAACAATGCCATGT
Mouse IL-1*β*	GCAACTGTTCCTGAACTCAACT	ATCTTTTGGGGTCCGTCAACT
Mouse IL-6	CTGCAAGAGACTTCCATCCAG	AGTGGTATAGACAGGTCTGTT
Mouse IL-18	GACTCTTGCGTCAACTTCAAGG	CAGGCTGTCTTTTGTCAACGA
Human *β*-actin	CATGTACGTTGCTATCCAGGC	CTCCTTAATGTCACGCACGAT
Human IL-1*β*	GTCGGAGATTCGTAGCTGGAT	CTCGCCAGTGAAATGATGGCT
Human IL-6	TGAGGAGACTTGCCTGGTGAA	CAGCTCTGGCTTGTTCCTCAC
Human IL-18	TCTTCATTGACCAAGGAAATCGG	TCCGGGGTGCATTATCTCTAC

## Data Availability

The datasets used and/or analysed during the current study are available from the corresponding author on reasonable request.
